The article "Vision-Based Intelligent Perceiving and Planning System of a 7-DoF Collaborative Robot" was published in 2021. Journal: Comput Intell Neurosci.

# Vision-Based Intelligent Perceiving and Planning System of a 7-DoF Collaborative Robot

**DOI:** 10.1155/2021/5810371

**Published:** 2021-09-14

**Authors:** Linfeng Xu, Gang Li, Peiheng Song, Weixiang Shao

**Affiliations:** ^1^Department of Mechanical & Aerospace Engineering, University of Florida, Gainesville 32611, FL, USA; ^2^Center Research Institute, SIASUN Robot & Automation Co. Ltd., Shenyang 110169, China; ^3^AI Robot Research Group, Peng Cheng National Laboratory, Shenzhen 518055, China; ^4^Research Department, FIFAN Robot Co. Ltd., Shenyang 110101, China

## Abstract

In this paper, an intelligent perceiving and planning system based on deep learning is proposed for a collaborative robot consisting of a 7-DoF (7-degree-of-freedom) manipulator, a three-finger robot hand, and a vision system, known as IPPS (intelligent perceiving and planning system). The lack of intelligence has been limiting the application of collaborative robots for a long time. A system to realize “eye-brain-hand” process is crucial for the true intelligence of robots. In this research, a more stable and accurate perceiving process was proposed. A well-designed camera system as the vision system and a new hand tracking method were proposed for operation perceiving and recording set establishment to improve the applicability. A visual process was designed to improve the accuracy of environment perceiving. Besides, a faster and more precise planning process was proposed. Deep learning based on a new CNN (convolution neural network) was designed to realize intelligent grasping planning for robot hand. A new trajectory planning method of the manipulator was proposed to improve efficiency. The performance of the IPPS was tested with simulations and experiments in a real environment. The results show that IPPS could effectively realize intelligent perceiving and planning for the robot, which could realize higher intelligence and great applicability for collaborative robots.

## 1. Introduction

An intelligent robot system should have the ability to interact with humans and environment, thus realizing collaboration and work with humans. Therefore, object grasping is one of the most important and significant abilities which could lead the robot to bring productivity to the society [1]. The robotic system for grasping is mainly composed of the perceiving system and the planning system. In existing applications, humans take great responsibility for perceiving and planning for robots as well as controlling them through computer programs. To truly realize intelligent working and collaborating, the “eye-brain-hand” process similar to humans has become an important researching field. However, intelligence leads to much higher requirements, and thus deep learning and data sets are designed and used to improve the ability of the “brain.” Thus, for wider application of collaborative robots, the ability to learn and then independently solve tasks based on a data set is more important and urgent than moving the robot to the perceived pose.

The article "Vision-Based Intelligent Perceiving and Planning System of a 7-DoF Collaborative Robot" was published in 2021. Journal: Comput Intell Neurosci.

Intelligent perceiving process has been studied for a long time, and many studies and products to support the perceiving system are realized. The performance and quality of perceiving received much attention, especially for 3D objects. Furthermore, the 6-DoF grasping means the object could be grasped from any angle in the 3D working space. With modern vision devices, such as Microsoft Kinect and Intel RealSense, more information of the objects in the working scene could be obtained easily through perceiving systems. The depth-based 6-DoF grasping methods lead the research direction, and most of them are focused on 6D object pose perceiving [2, 3]. Researchers also focus on the combination with deep learning to further improve intelligent perceiving [4, 5]. The visual process of intelligent perceiving is also important for the performance of the whole system. For 3D object visual process, existing methods include random sample consensus (RANSAC) [6], Hough-like voting [7], and FPFH [8]. Rabbani realized an efficient Hough transform for automatic perceiving of cylinders. Rusu realized the visual process in the segmented scenes and used triangular meshes to create a hybrid shape-surface for robotic grasping. In this research, considering the type of the feature, a combination of FPFH method and ICP algorithm, which effectively improved the speed and accuracy of the registration compared to common registration method, was designed.

Based on the perceiving process, many data sets have been established, which greatly show the development of intelligent and deep learning. Representative data sets include PASCAL VOC [9], SUN [10], ImageNet [11], MS COCO [12], and Open Images [13]. These data sets could be used to train the network to predict the bounding box and precise grasping points of the object. Some famous grasping data sets have been appeared in a great number of research works, such as Stanford grasping data set, Cornell grasping data set, YCB benchmarks data set, CMU data set, Google data set, Dex-Net 1.0, Dex-Net 2.0, and JACQUARD. Besides, grasping planning data sets receive much attention from researchers. Pinto and Gupta proposed a data set size of 50K data points which collected 700 hours of grasping attempts [14]. Levine realized 800,000 grasp attempts in two months [15]. Wang realized a visual-tactile grasping data set with a dexterous robot hand by Intel [16]. Andrew and Peter proposed GraspIt! containing a simulator for robotic grasping to interactively manipulate a robot [17]. Quillen proposed a simulated grasping benchmark for the manipulator [18].

The article "Vision-Based Intelligent Perceiving and Planning System of a 7-DoF Collaborative Robot" was published in 2021. Journal: Comput Intell Neurosci.

Intelligent planning for robot system has always been a hot topic for researchers. 3D object planning is based on accurate prediction including object prediction or detection, grasping position prediction, and grasping point prediction. The prediction of the 3D bounding box of the object is an important step for intelligent planning. The 3D bounding box prediction is similar to 6D object pose prediction. Methods of 3D visual process could be used here, such as FPFH [8], CVFH [19], SHOT [20], and ICP [21], which can locate the object and realize registration for the object. Deep learning could make the prediction more efficient and the bounding boxes could be predicted with features extracted from neural network. Frustum PointNets realized 2D CNN prediction and lifted the 2D region to a 3D region [22]. PointFusion used Faster RCNN [23] to obtain the deep features from the image to build the 3D bounding boxes [24]. Frustum ConvNet also obtained the 3D region through lifting the 2D region [25]. Methods based on global features require enough input to generate the region. Deep Sliding Shape was the first 3D region prediction network (RPN) using CNN, which could extract geometric features and color features in 2D to predict the bounding boxes [26]. Real-time prediction of the 3D region with motion parameters for unknown moving object was a further research topic [27]. In this research, a new CNN was designed to realize grasping region planning through lifting a bounding box from rectangle predicted with the input images, which could effectively improve the speed and accuracy of the CNN with less parameters and information needed. 3D object bounding box prediction is not accurate enough to realize grasping planning for the robot hand, but it could provide a proper and general grasp position for further planning of grasping contact points.

The grasping position and grasping point planning or prediction are crucial for intelligent planning, which could improve the performance and collaboration ability of the robot greatly. Empirical method is a data-driven method to learn from successful results and plan to grasp objects, which can solve the grasping of known or unknown object [28]. Miller proposed a method to classify objects into categories corresponding to grasping types [29]. Vahrenkamp divided objects based on geometric information and labeled information [30]. It is hard for the grasping planning based on a data set to grasp the unknown object. Therefore, in this research, an operation recording set was established as grasping experience could effectively solve this problem. Mahler established a grasping data set with the depth image and many object grasping points, which has more than 50k grasps, and the grasping performance was great [31]. The grasping points could be directly predicted from the input image only. Pinto and Gupta proposed a method to predict grasp locations with a CNN-based classifier to predict the grasp [14]. Park proposed an accurate grasping prediction method with fully CNN to obtain the poses for the manipulator [32]. Zeng designed a multi-affordable planning method to select the grasping types and recognize the object in product images [33]. In this research, a new CNN was designed together with grasping type to realize grasping point planning based on the bounding box planning and well-designed calculation, which could greatly improve the speed, accuracy, and success rate of the CNN and realize higher intelligence.

The article "Vision-Based Intelligent Perceiving and Planning System of a 7-DoF Collaborative Robot" was published in 2021. Journal: Comput Intell Neurosci.

The intelligent planning process contains an important part which is the trajectory planning for the manipulator. Through imitation learning, deep learning could learn from successful grasping attempts in the data set and finish grasping with a movement similar to human operation. Amor realized imitation learning to achieve grasping ability based on human operation [34]. Ebert tried to learn robotic skills from images from observations of collected experience to realize planning for unlabeled data [35]. Fang realized a task-based grasping planning network when being input by the vision system [36]. Wu realized coordinated planning of a dual-arm robot for surgical instrument sorting tasks [37]. Many traditional planning algorithms have been proposed worldwide, including ant colony algorithm [38], LPA∗ algorithm [39], D∗ Lite algorithm [40], and PRM algorithm [41]. The traditional trajectory planning method is suitable for the working space where the obstacle position is determined and ensures high efficiency and accuracy. Rapid random tree RRT algorithm could plan the trajectory through random sampling, which fits the trajectory planning of 7-DoF robots with infinity mobility in high dimensional space [42]. To solve the shortage of RRT like low speed for large environment, improved RRT algorithms have been proposed. The bidirectional RRT sets the steps from the terminating and starting point at the same time [43]. In this research, an improved trajectory planning algorithm was proposed; it combined interpolation with RRT algorithm with the operation recording set to improve the collaboration ability and man-robot interaction performance.

The article "Vision-Based Intelligent Perceiving and Planning System of a 7-DoF Collaborative Robot" was published in 2021. Journal: Comput Intell Neurosci.

In this research, a new system based on deep learning, known as IPPS, was proposed and implemented to realize intelligent perceiving and planning for robot hand and manipulator. The most important innovations and contributions of IPPS are as follows. First, a new operation and environment perceiving process was proposed, including a well-designed vision system, a new hand tracking method, and fingertip marking. Then, a new operation recording set was established based on the perceived operation process and daily object data set. Besides, a new grasping and trajectory planning method was proposed based on the deep learning with CNN and the operation recording set to realize grasping gesture type prediction, grasping bounding box prediction, and contact point prediction for three-finger robot hand. Finally, a new trajectory planning method for the manipulator which combined interpolation based on the operation recording set and the tracking records of the vision system with RRT algorithm was proposed. IPPS was tested with simulations for every new method and algorithms and application in real environment for its efficiency, accuracy, and stability, which could effectively realize the intelligence perceiving and planning of the robot and achieve higher collaboration ability and better man-robot interaction.

### 1.1. Intelligent Perceiving Process

The most convenient way to achieve the intelligence of the robot is learning from human operation experience. However, the existing data sets mainly contain object images only and lack records of operation, which could make it difficult for the robot to gain sufficient experience. To solve this problem, establishing an operation recording set is necessary. The main process contains two parts: one is recording the human hand operation process, and the other is tracking the marked hand posture at the same time. Besides, the vision system can also perceive the environment when IPPS is applied to the robot to start the whole process. The perceived image could be used as the input to the neural network for deep learning to realize planning. Intelligent perceiving is acting as the “eyes” for the robot to observe human operation for learning as well as the objects and tasks for planning the man-robot interaction.

#### 1.1.1. Vision System with Cameras

The completeness of operation data and object and scene images is important for the performance of perceiving. Therefore, in addition to two three-dimensional RGB cameras as the binocular fixed vision system, an eye tracker is designed as the follow-up vision system in this research, which could be worn by the operator when operating. Besides, environment perceiving will be finished with another depth camera on the top for registration and trajectory recording. The entire vision system is shown in Figure 1.

The article "Vision-Based Intelligent Perceiving and Planning System of a 7-DoF Collaborative Robot" was published in 2021. Journal: Comput Intell Neurosci.

Compared with a single fixed vision system, the combined vision system could observe the hand motion and the marked points from adjustable and different angles as the eye tracker could finish real-time following and achieve images from several directions to reduce data loss caused by occlusion. All images achieved from the vision system could be saved to the operation recording set. For environment perceiving, the fixed cameras from different angles could make sure that the observation is comprehensive and provide enough information in the images for the neural network to plan for the operation of robot. The vision system is combined with operation perceiving and environment perceiving camera system. These two camera systems work separately in the whole IPPS at different steps when realizing the robot but they share much information together to support higher intelligence for the robot. The complete information achieved from the vision system could provide great support for operation recording set establishing and intelligent robot planning.

#### 1.1.2. Hand Posture Tracking

The establishment of a data set for hand operations is crucial for further deep learning. Some methods have been proposed like using marked gloves which limit the flexibility of the hand and affect the data. When a human grasps an object, the operation is usually hard to track with plenty of movable joints. Therefore, in this research, a new method to realize hand tracking was proposed to achieve finger joint angles and hand posture effectively. Considering that most parts of the hand deform when grasping, the fingertips of the thumb, index, and middle finger could not be easily affected, and the corresponding position could represent the contact points on object at the same time. If the positions of three fingertips and wrist could be confirmed, the joints of every finger and the hand posture could be obtained through analysis of kinematic constraints. The hand structure is shown in Figure 2.

In this research, the robot hand designed mainly includes proximal phalanx, middle phalanx, and distal phalanx, in addition to four types of joint points: MCP (metacarpophalangeal), PIP (proximal interphalangeal), DIP (distal interphalangeal), and IP (interphalangeal). The relationship is shown in (1) and (2). The constraints are necessary because they are the natural relations between joints, which can make the robot hand similar to the human hand and achieve better grasping performance.

(1) $$\begin{array}{c} \theta_{\text{DIP}}\approx \frac{2}{3}\theta_{\text{PIP}}\theta_{\text{PIP}}\approx \frac{3}{4}\theta_{\text{MCP}}, \end{array}$$

(2) $$\begin{array}{c} \theta_{\text{IP}}\approx \frac{1}{2}\theta_{\text{MCP}}. \end{array}$$

Constraints also exist between two joints of different fingers. For example, when bending the index finger at the MCP, the MCP of the middle finger will bend at the same time. The relationship between the index and middle fingers when the index finger MCP is flexed is shown in the following equation:

(3) $$\begin{array}{c} \theta_{{\text{MCP}}_{\text{middle}}}\approx \frac{1}{5}\theta_{{\text{MCP}}_{\text{index}}}. \end{array}$$

Besides, to reduce the difficulty of kinematics analysis, the robot hand will keep only the necessary DoF for grasping with three fingers. Considering the limited mobility, the solution will be single and solvable for the fingers and thumb. The forward and reverse kinematics can be easily solved through D-H method with MATLAB and robotics toolbox. The fingertips can be achieved by perceiving and represent the contact points on the object. The error of reverse kinematics is evaluated with standard deviation which is set to be less than 0.1 to ensure the effectiveness of the new hand tracking method.

The article "Vision-Based Intelligent Perceiving and Planning System of a 7-DoF Collaborative Robot" was published in 2021. Journal: Comput Intell Neurosci.

#### 1.1.3. Operation Recording Set Establishment

In this research, operation recording set of different representative objects could ensure that the data set has great applicability. Unlike the data set with only object images, the operation recording set could be a solid foundation for further deep learning and planning, which could make the manipulator and the robot hand achieve the experience of human operation and finish grasping more similar to human arm motion and hand grasping gesture.

The establishment of the recording set mainly includes two steps: one is recording the human operation, and the other is operation data processing. The vision system records the marked point information when a human is operating and grasping the objects completely. The recording of the operation process is shown in Figure 3. In this research, 24 objects were used to ensure the effectiveness of the operation perceiving, and RGB images were recorded for different operation types for each object. The operation recording set could effectively bring better applicability, as deep learning could achieve the experience from human operation, which results in better performance in man-robot interaction in real applications.

#### 1.1.4. Environment Perceiving and Visual Process

The environment perceiving is also important to the intelligent perceiving process, especially the manipulator. Depth camera at the top could realize the registration and positioning of the object at the beginning. However, with the existence of interference like noise and other factors, the images and data acquired need a proper visual process to improve the quality. The visual process starts with filtering and top point cloud obtaining. Point cloud filtering is realized through calculating the average distance of all threshold neighbor points and eliminating the terrible points. Obtaining the top point cloud is to obtain the highest *z*-direction layer of the remaining point cloud as the feature of the object to reduce the difficulty of registration.

The article "Vision-Based Intelligent Perceiving and Planning System of a 7-DoF Collaborative Robot" was published in 2021. Journal: Comput Intell Neurosci.

The registration is realized with coarse registration and accurate registration. The coarse registration can make the actual object be basically matched with the object in the data set. In this research, FPFH was used, which is realized based on the feature histogram. The principle used is the sampling consistency method. Then, the accurate registration can make the object and the model accurately registered. In this research, ICP algorithm was used, which is based on calculating and evaluating the sum of the squares of the Euclidean distance between all corresponding points as in the following equation:

(4) $$\begin{array}{c} f\left(R,T\right)=\frac{1}{N_{P}}\sum_{i=0}^{N_{P}}{\left|p_{t}^{i}-R\cdot p_{s}^{i}-T\right|}^{2}, \end{array}$$

*p* is the corresponding points and *N* is the total pairs. Besides, *R* and *T* are rotation and translation matrix, respectively. A confidence threshold is needed for evaluating the registration, which was set to be higher than 97%. The registration is shown in Figure 4.

### 1.2. Intelligent Planning Process

The robot hand has a structure similar to the human one, so it potentially has great collaboration ability and may even replace human hands in some specific environments and tasks. Therefore, to realize collaboration in more scenes and conditions, an intelligent planning method was proposed in this research, which includes simple object-based grasping planning and complex task-based operation planning. By adding the trajectory planning of the manipulator, the intelligent planning system for the robot could be realized completely. The data obtained through the perceiving process could be used by the neural network, and it could get a basic command of human operation, to realize intelligence planning when being given objects or tasks through the environment perceiving like humans.

#### 1.2.1. Grasping Region Planning

In this research, grasping region prediction from RGB images of the object in the working scene is an important task. The performance of grasping is judged by the success rate and error of pose. A successful grasping process is considered when the object is truly grasped, held, and moved to realize man-robot interaction tasks. A grasping region rectangle can be described as follows:

(5) $$\begin{array}{c} g\left\{x,y,h,w,\theta \right\}, \end{array}$$

where *x* and *y* describe the center of a rectangle grasping region; *h* and *w* describe its size in terms of height and width; and *θ* describes the orientation relative to the horizontal axis of this image. The example of this representation is shown in Figure 5(a). This representation works well in practice as it expresses the grasping in the coordinate system of this image. Based on the rectangle grasping region with *x*, *y* position, the *z* position could be described as the depth and the distance which is vertical to the image. Therefore, if using two RGB images from different angles could achieve the depth and distance, the rectangle could be lifted along its depth to get a 6D grasping region, a bounding box, as shown in Figure 5(b).

The article "Vision-Based Intelligent Perceiving and Planning System of a 7-DoF Collaborative Robot" was published in 2021. Journal: Comput Intell Neurosci.

When performing the grasping method on the real robot, *h*, *w*, and *d* bound the robot hand. Moreover, compared with traditional six-dimensional grasping based on point cloud, the grasping box achieves the location and orientation based on five-dimensional grasping rectangle and depth, which will reduce the calculation and save a great deal of time for the neural network to train and learn. The CNN for six-dimensional grasping box planning is shown in Figure 6. The CNN extracts the global and local features to plan. For example, if the object is an apple, the global features give shape information that the object is most likely to be an apple. Therefore, the position of the grasping should be the circle near its top. Besides, the local features give the edge, which provides the contact region. Finally, the last fully connected layers could save the training time greatly and output the parameters.

A threshold is used to consider the success of grasping planning. The rectangle region of grasping is used for evaluation, and a grasp is considered successful, good, or correct if the difference between the predicted angle and true angle is less than 30 degrees and the Jaccard index of the predicted grasp and true grasp is more than 25%, which is defined as follows:

(6) $$\begin{array}{c} J\left(\hat{\theta },\theta \right)=\frac{\left|\hat{\theta }\cap^{}\theta \right|}{\left|\hat{\theta }\cup \theta \right|}, \end{array}$$

where *θ* hat is the predicted grasp and *θ* is the truth grasp, which represents the ratio of the overlapping to the total. For all objects in the data set, the best scored grasp rectangles using the planning method are selected. Combined with the end pose of the manipulator, the grasping gesture can be totally decided. However, even though planning for the bounding box can solve most grasping problems, it actually supports the grasping with gripper. The planning for a complex and accurate task needs better flexibility of grasping. Therefore, the fingertips position is important information to realize truly intelligent grasping planning.

The article "Vision-Based Intelligent Perceiving and Planning System of a 7-DoF Collaborative Robot" was published in 2021. Journal: Comput Intell Neurosci.

#### 1.2.2. Contact Point Planning

Intelligent collaboration has higher requirements for grasping planning. When humans grasp objects, the gestures of the hand could be mainly divided into some certain types, and the ones fitting with three-finger robot hand are large wrap, medium wrap, small wrap, adducted thumb, power sphere, tripod, lateral pinch, and two-finger-thumb precision. A simple CNN was designed for grasping gesture prediction with object images input. The grasping type and the grasping region are both necessary to realize independent control of each finger. Therefore, another CNN was proposed in this research. If the end pose of the manipulator could represent the gesture of the wrist of the robot hand and the position of the fingertips could represent the contact points, the pose of every finger joint can be calculated, hence the intelligent control of the hand. The CNN for contact point planning is shown in Figure 7.

CNN is used to extract the features of the object with four convolution layers to describe the object combining with the grasping type. Therefore, if the object is an apple this time, the global features show that the object could be an apple and so the basic grasping position is determined. The local features give the edge information for the grasping rectangle planning. With double RGB images input, the depth can be used to translate the rectangle to form a grasping box, which could totally limit the grasping region. Finally, the gesture type based on the thumb pose type is input to finally decide the accurate contact points. The contact points for three fingers could be calculated as follows:

(7) $$\begin{array}{c} {\text{cp}}_{\text{thumb}}=\left(x-\frac{w}{2}\cos\theta ,y+\frac{w}{2}\sin\theta ,z+\frac{d}{2}\right), \end{array}$$

(8) $$\begin{array}{c} {\text{cp}}_{\text{finger}}=\left(x+\frac{w}{2}\cos\theta \pm \frac{h}{2}\sin\theta ,y-\frac{w}{2}\sin\theta \;\mp \;\frac{h}{2}\cos\theta ,z+\frac{d}{2}\right), \end{array}$$

where cp is the contact point position, (*x*, *y*, *z*) is the image center, and (*w*, *h*, *d*) is the box size. It can be assumed that high-quality grasps are achieved when the geometric center of the box or the rectangle which is formed with three fingertips is located near the true geometric center of the object. Therefore, we assign the geometric center score to describe the distance from the grasping points related to the geometric center of the object, thus evaluating the quality of the contact points as follows:

(9) $$\begin{array}{c} c_{gc}=\frac{d_{\max}-d}{d_{\max}-d_{\min}}, \end{array}$$

where *c*_*gc*_ is the geometric center score, *d* is the distance from the center of grasping points to the geometric center of the object, and *d*_max_ and *d*_min_ are the maximum and minimum distance between any grasping point center planned and the corresponding object geometric center. The error of grasping point planning is evaluated with MSE which is set to be less than 2.5, and the success rate is set to be higher than 85% to ensure the accuracy and effectiveness of the new CNN proposed.

The article "Vision-Based Intelligent Perceiving and Planning System of a 7-DoF Collaborative Robot" was published in 2021. Journal: Comput Intell Neurosci.

In real life, when dealing with a cup, the collaboration is not only grasping the cup, but moving to the human, removing the closure, or pouring out, which requires the high complexity and intelligence of robot. This CNN can effectively realize the accurate grasping task with independent finger controlling. When the object in its scene is perceived, classified, and positioned with the vision system, the grasping type and grasping region on a cup will be planned if the object matches the data set well. The grasping will be realized, and the manipulator could finish the task and realize man-robot interaction, thus achieving higher intelligence to the robot.

#### 1.2.3. Manipulator Trajectory Planning

The trajectory planning of the manipulator is another part of the planning in this research. Traditional trajectory planning methods mainly solve the joint angle of a manipulator from the starting pose to the end pose through reverse kinematics. However, the reverse solution of multi-degree-of-freedom manipulator like 7-DoF manipulator is uncertain and could not conform to the optimal trajectory.

The operation recording set has been established during the perceiving process, which could record the operation process, which could be used for the whole trajectory perceiving. The marked information of the hand in each image could be used to improve the trajectory planning. For the 7-DoF manipulator, it is more efficient to plan for the end pose. In this research, the intelligent trajectory planning method was combining RRT with interpolation as the records could make it much more convenient to interpolate points and lead the manipulator to move as a human arm. The flow chart of the interpolation with RRT is shown in Figure 8.

To estimate the quality during the trajectory planning of the manipulator, the end pose of the manipulator is used to check the pose error. The pose can be represented by a 4 × 4 matrix *P* = [*R*, *t*], where *R* is a rotation matrix and *t* is a translation vector. Based on the forward and reverse kinematics of the 7-DoF manipulator, the relationship of the joint angle and end pose can be used to correct the trajectory and evaluate the performance as follows:

(10) $$\begin{array}{c} R^{\text{error}}=R^{T}R^{\text{ref}}, \end{array}$$

(11) $$\begin{array}{c} t^{\text{error}}=t^{\text{ref}}-t, \end{array}$$

(12) $$\begin{array}{c} \text{error}={\left|t^{\text{error}}\right|}^{2}+{\left|\omega^{\text{error}}\right|}^{2}. \end{array}$$

The error is dependent on the translation vector *t* and angle vector *ω* from the rotation matrix *R*. The error of trajectory planning is set to be less than 2.5%, and the efficiency is evaluated with the trajectory length and planning time compared to the traditional RRT to ensure higher accuracy and efficiency of the improved RRT proposed. The error of the trajectory planning is important as the grasping planning needs the accurate end pose of the manipulator or the success rate will be uncontrollable and meaningless. The performance of trajectory planning could improve the quality of intelligent planning process and the ability of man-robot interaction for the collaborative robot.

The article "Vision-Based Intelligent Perceiving and Planning System of a 7-DoF Collaborative Robot" was published in 2021. Journal: Comput Intell Neurosci.

## 2. Results and Discussion

In this research, IPPS was verified in terms of the perceiving process, the planning process, and the whole system application to the robot. The verification was composed of simulations and experiments in a real environment. The simulation platform used in the research was MATLAB. The industrial computer was configured as NVIDIA RTX3080 and Intel Core i9-11800H @ 2.3 GHz, and the memory was 32 GB. The experiments in the real environment were realized based on the hardware system including SCR5 manipulator and Mech III robot hand. Xbox One Kinect camera, Intel RealSense D415, and Microsoft HoloLens 2 were used for perceiving. The experiments comprehensively ensure the effectiveness and intelligence of the IPPS for the collaborative robot.

### 2.1. Intelligent Perceiving Process

In this research, the vision system was built up for intelligent perceiving. The perceiving process is not only used to perceive the environment to finish the tasks but also to perceive and record the objects as well as the operation to establish the recording set for deep learning and intelligent planning. Actually, the intelligence of IPPS is mainly based on a well-designed data set with different types of objects and some corresponding operations in daily life. In this research, the images of objects and operation were recorded and marked information was stored, thus realizing further intelligent planning. Moreover, the perceiving of the operation is important for manipulator trajectory planning. The visual process of the perceiving process influences a lot the quality and accuracy. The effectiveness and rationalization of the perceiving method and the recording set establishment as well as the stability and accuracy of the marking and tracking method were tested. Besides, the accuracy and stability of the visual process were tested to evaluate the environment perceiving.

The article "Vision-Based Intelligent Perceiving and Planning System of a 7-DoF Collaborative Robot" was published in 2021. Journal: Comput Intell Neurosci.

#### 2.1.1. Vision System for Perceiving

The perceiving process is realized based on a well-designed vision system. The perceiving of human hand operation is one of the main parts of perceiving as well as the starting point of IPPS. In this research, the double fixed RGB camera group and a tracking vision as an eye tracker worked together as the new vision system of operation perceiving, as shown in Figure 9(a). The environment perceiving for the application was realized by the combination of the depth camera on the top and two RGB cameras in front of the working scene, as shown in Figure 9(b). The depth camera could realize registration and positioning to trigger the whole process and reduce the use of deep learning. Moreover, the recording could be of great importance to the trajectory planning.

When realizing the application of IPPS to the robot and manipulator, the environment perceiving was realized first with two steps. First, the depth camera perceives the environment first to match the object and get the position information from the visual process. If the object was matched, the RGB cameras would perceive the environment and get the accurate feature and pose information for deep learning. The environment perceiving is shown in Figure 10.

In the research, the real environment with a working scene like a table, with many daily objects at different poses on it, could be messy and difficult to perceive. The combined camera system could make it more comprehensive to perceive the scene and get more information. A table was placed with different combinations of several objects to build up different kinds of daily scene of the table. The well prepared and designed objects' kind and working scene could greatly influence the quality and applicability of the system.

#### 2.1.2. Hand Tracking and Marking

Tracking and marking of the hand are crucial for recording sets. In this research, the effectiveness of the new method of hand tracking and finger joint angle achieving was tested and verified. Three different colored tapes in red, yellow, and blue were tied on the thumb, index, and middle fingertips, respectively, as shown in Figure 11(a). In this research, the robot hand was designed based on the proximal phalanx, middle phalanx, and distal phalanx with four joint points: MCP, PIP, DIP, and IP, as shown in Figure 11(b).

The article "Vision-Based Intelligent Perceiving and Planning System of a 7-DoF Collaborative Robot" was published in 2021. Journal: Comput Intell Neurosci.

The joint angles of three fingers were calculated based on the kinematic constraints relationship, and the reverse kinematics was realized with MATLAB. There is only one solution for the thumb as it is a 3R mechanism. However, there are two solutions for the index and middle finger as they are 4R mechanism and the mobility is 1. The optimal solution was the one with positive angle change for DIP and IP. The hand posture calculation was tested with 4 grasping types, respectively, and 5 tests each with the manipulator reaching the grasping point. The results of reverse kinematics tests are shown in Table 1. It could be seen that the solutions obey the kinematic relationship and effectively finish grasping with a standard deviation of joint angles less than 0.05. The stability and accuracy of kinematics could ensure the precise grasping as well as the application value of the recording set.

#### 2.1.3. Visual Process

The visual process for intelligent perceiving is an important step for the whole system. The object data set in this research was designed with the top layer model perceived from the depth camera, as a vision from the top could set up a model with less data than the front vision system, which could effectively reduce the calculation for registration. The registration of the object had two steps: first coarse registration based on FPFH and then use of ICP algorithm to modify and finish the accurate registration. The registration performance was tested with 22 objects in this research, and the accuracy of translation and rotation and confidence of registration were used for evaluation. The results are shown in Figure 12.

It shows that the accuracy of registration is 98.85% on average, and the confidence of registration is 99.45% on average, which could effectively ensure the quality of the visual process. Objects without a typical top layer have lower registration confidence and accuracy because of the characteristic of depth camera. For example, when matching an object such as a cup in the scene, the registration with other objects such as metal can and small bowl could also exceed the confidence threshold to make a confusion. Thus, two-step registration is needed to realize the better performance of environment perceiving. Based on the tests for the objects, the accuracy and confidence are enough for the intelligence requirements and could greatly support the planning process and improve the performance of the IPPS.

### 2.2. Intelligent Collaboration Planning

The new intelligent planning method proposed aimed at achieving better collaboration ability through realizing higher intelligence of robot. In this research, the performance of the new intelligent planning method for robot hand based on deep learning and trajectory planning for manipulator based on the combination of RRT and interpolation were tested. The experiments mainly checked the effectiveness of gesture type prediction, and the accuracy and stability of grasping box and grasping point prediction. Besides, the accuracy and efficiency of trajectory planning were also tested. Finally, the performance of the intelligent planning process and the IPPS was tested in a real environment. The simulation and experiments with the robot could ensure the effectiveness and stability of IPPS and show the performance and value of the intelligent system, which could realize intelligence perceiving and planning as well as man-robot interaction for collaborative robot.

The article "Vision-Based Intelligent Perceiving and Planning System of a 7-DoF Collaborative Robot" was published in 2021. Journal: Comput Intell Neurosci.

#### 2.2.1. Grasping Gesture Prediction

The gestures of grasping were divided into eight types for the three-finger robot hand. Deep learning was used to plan for the grasping gestures. A CNN neural network was designed with the object RGB images from the perceiving process as the input and the grasping type as the output. Based on deep learning with the network, the performance of grasping gesture prediction with different objects was tested with five selected objects: noddle box, tea cup, coke bottle, tape, and apple. The success rate and speed are shown in Table 2.

The speeds shown in this table were the average of the prediction speed of every test for each object selected. The success rate here is to evaluate the matching of the predicted type and the object. Object 3, which is the coke bottle, is the one that leads to the best results in both the success rate and speed. However, object 2, which is the tea cup, has the worst performance, and this condition suggests that the number of local features and the complexity of global features will influence the CNN extracting quality for prediction and thus the grasping gesture. Based on the grasping gesture, the robot can solve simple grasping problems and even similar objects with the same features as the objects in the data set.

#### 2.2.2. Grasping Position Prediction

The grasping position prediction of the object is important for intelligent planning, which could be evaluated with the success rate and error of position. The method proposed in this research was based on deep learning. The input of the RGB images could realize a rectangle grasping region prediction and supply the information of distance, position, and thus depth. The depth was then combined with the predicted rectangle to find a bounding box, which bounded and limited the robot hand grasping position, and realize intelligent grasping.

The article "Vision-Based Intelligent Perceiving and Planning System of a 7-DoF Collaborative Robot" was published in 2021. Journal: Comput Intell Neurosci.

The grasping box predicted for the objects and combinations is presented in Figure 13, which directly shows the stability and effectiveness of the prediction method adapting to different shapes, sizes, and poses. It can also be seen that some special cases show more of this network. The objects in Figures 13(a) and 13(c) are easier for the network to predict as they are mostly standing in the scene with a proper thickness. Most objects like these allow a good grasping prediction. The objects in Figures 13(d) and 13(e) are laid, which makes it a bit hard to predict the box. The tea cup in Figure 13(b) presents a higher challenge, as it contains several features leading to multiple grasping positions. It could be noted that the CNN for grasping region prediction has the ability to make intelligent choices. The performance of the CNN was tested with three combinations as shown in Figure 13(f). It could be seen that the presence of multiple objects did not influence the stability of the network.

The threshold used to evaluate the success of grasping position planning was the error of the bounding box with the angle and the rectangle relation, as the depth is accurate enough based on the binocular mechanism. Five selected objects were used to test the performance of the network in terms of accuracy, speed, and success rate. The best grasp rectangle using the planning method was considered, and the results are shown in Table 3.

The performance is tested with a success rate based on the threshold, and the error of the prediction is based on the successful grasping. Therefore, the high success rate could also support the evaluation of the prediction performance. Object 3 shows the best results in the success rate and error. Object 1 leads the best speed performance based on its obvious depth. Object 2 shows the lowest speed as well as the highest error, which could illustrate the influence of the shape complexity and task combination on the CNN performance. The better grasping position prediction performance could make the planning of grasping points much easier and effectively improve the accuracy of the whole grasping planning.

#### 2.2.3. Grasping Point Planning

Independent control of each finger is necessary for intelligent grasping planning, to reduce the calculation pressure for deep learning as there are too many parameters for hand pose information. Therefore, the grasping points or the contact points on the object are important to solve the control of three fingers. The CNN proposed in this research could realize contact point planning as shown in Figure 14.

The article "Vision-Based Intelligent Perceiving and Planning System of a 7-DoF Collaborative Robot" was published in 2021. Journal: Comput Intell Neurosci.

In Figure 14, eight prediction examples are shown, including the five selected objects and three combinations to show the effectiveness of the grasping point prediction. The objects contain complex features and different sizes and poses, which can ensure the applicability in real scenes. The tea cup still poses a challenge. The CNN predicts the gestures required for grasping the cup and moving it, so the grasping points are proper. If the task changes to grasping the handle, the prediction will be much harder. Totally, the grasping point prediction could effectively realize intelligent grasp planning. The performance was also tested with three combinations as shown in Figures 14(f)–14(h), which ensures the stability and effectiveness of the method.

The quality evaluation of grasping point prediction was based on the error of the position. Assuming that the mass of the object is uniformly distributed for most daily objects, a bottle of water will be a considerable problem. Therefore, the difference between the geometric center of the object and the center of three grasping points was used. Besides, the success rate was based on whether the predicted three grasping points could truly realize the grasping. The five selected objects were used to test the performance of the network in terms of accuracy, speed, and success rate as shown in Table 4.

It could be seen from the table that object 3 leads in the speed, success rate, and error, which ensures great intelligence and accuracy for grasping planning. Objects 1 and 5 also perform well. Objects 2 and 4 have a bit larger error and lower success rate as the complex shape influences the grasping position prediction. The accuracy and the success rate could prove that the grasping planning process could effectively and accurately realize intelligent planning for the robot hand. When dealing with a cup, the collaboration is not only grasping the cup, but moving to the human, removing the closure, and pouring out as well. These tasks are combined with grasping points and object features. If the task is taking the cup to the human or pouring the water, the grasping points need to be planned. However, features like body and handle can realize grasping, moving, and pouring. Decision and planning lead to high complexity of intelligence and thus influence the requirement for the ability of the CNN.

#### 2.2.4. Trajectory Planning

The trajectory planning of the manipulator is the final step of intelligent planning. To solve the reverse kinematics problem of 7-DoF manipulator, the new trajectory planning method was proposed to combine interpolation with RRT. This method could plan for the trajectory similarly to human arm operation with less time and better end pose translation. The tests were set up for five selected models beginning at the origin pose, where all joint angles of the manipulator were zero. The objects were placed in the working space of the manipulator and perceived with the vision system to get the information, which would be the final pose or the desired pose of the manipulator. The differences between the achieved pose through planning and the desired pose by perceiving are presented in Table 5.

The article "Vision-Based Intelligent Perceiving and Planning System of a 7-DoF Collaborative Robot" was published in 2021. Journal: Comput Intell Neurosci.

The accuracy of position and orientation shows the ability of the trajectory planning method to realize the intelligent planning for the manipulator. The effectiveness of trajectory planning mainly relies on good modeling and effective operation recording set as well as well-designed vision system. The trajectory planning method could obtain an accurate position with less than ten-millimeter error and less than one-degree orientation error. The performance of the trajectory planning method was also tested in 3D plots with occlusion in the scene with MATLAB, as shown in Figure 15.

It could be seen that the trajectory planning performs well for all objects with a proper motion path in 3D space because of the interpolation points from the operation recording set. It is obvious that the tree is more similar to a direct motion to the objects, especially when it is getting closer as the interpolation points were mainly set near the object. The RRT algorithm in this research also designed with collision detection and obstacle avoidance further improves the ability of trajectory planning as only moving the manipulator to the final point is meaningless for an intelligent collaborative robot. The accuracy, efficiency, and speed of the improved RRT compared with tradition RRT are shown in Table 6.

The interpolation affects the searching step length of RRT, thus influencing the efficiency and quality of planning. It could be clearly seen that, compared with traditional RRT, the improved RRT effectively reduces the trajectory length and planning error, especially the planning time, which could greatly improve the accuracy and efficiency of the trajectory planning. The performance quality of trajectory planning is so important that the grasping point planning is based on the accurate end pose of the manipulator and the success rate of IPPS application to real robot needs high quality of intelligent planning.

### 2.3. Experiments in the Real Environment

Finally, the performance of IPPS application to the collaborative robot was tested in a real environment. An object and its scene as well as the task were given; the intelligent perceiving process with the vision system started and the visual process including registration and positioning were finished. The central computer planned the trajectory of the manipulator with improved RRT through interpolation. An operation similar to human motion was predicted, and the manipulator was moved to the predicted pose. At the same time, the RGB images perceived were input to the CNN to plan the grasping points. TCP/IP realized the communication between the cameras, the computer, and the robot hand. The force sensor on the robot hand received the message of grasping, and if it succeeded, the computer would control the manipulator to move to the man-robot interaction position and finish the task. Finally, the manipulator and the robot hand will return to the origin pose. The process of IPPS application in real environment is shown in Figure 16.

The article "Vision-Based Intelligent Perceiving and Planning System of a 7-DoF Collaborative Robot" was published in 2021. Journal: Comput Intell Neurosci.

The performance of IPPS was tested with repeated experiments of different objects and different combinations; in particular, several groups of unknown objects were set to test the intelligence of the system. To ensure the effectiveness and stability of IPPS, 100 grasping attempts were considered for 14 representative single objects, 3 combinations, and 3 groups of unknown objects. The result of the experiments is shown in Table 7.

These results indicate a success rate of 87%; they contain thirteen failure cases with six of them due to neural network grasping prediction and seven of them due to trajectory planning. The excellent success rate could verify the stability and effectiveness of IPPS. The unknown object groups could evaluate the adaptation of the IPPS based on learning. It could be seen that the collaborative robot with IPPS successfully realizes the process of intelligent environment perceiving as well as trajectory and grasping planning. In addition, the performance of man-robot interaction is well enough for the intelligence requirements. IPPS has been fully verified with simulations and experiments in real environment, which has great application prospects for collaborative robots in the future.

## 3. Conclusions

This paper proposes an intelligent perceiving and planning system based on neural network, which could effectively realize the intelligence of collaborative robot. For the perceiving process, a vision system was built; a new method of hand tracking through marking the fingertips was proposed, and its effectiveness was tested with the accuracy of reverse kinematics; and an operation recording set was established to enhance collaboration ability through learning from the experience of human and achieving intelligence. The designed visual process was tested with objects to ensure the accuracy and stability of the environment perceiving. The planning process is based on deep learning. The new grasping planning method with CNN was proposed to find the contact points and tested, which could realize accurate and efficient planning for known and unknown objects to ensure the quality of intelligence planning for the robot hand. The new trajectory planning method for manipulator, which combined interpolation with RRT algorithm, was proposed. The tests show a reduction in planning length and time as well as the pose error which could supply higher accuracy and efficiency to the planning process. Finally, IPPS was tested in a real environment and could successfully realize intelligent perceiving and planning with high efficiency and stability that could meet the requirements of intelligence. IPPS could influence the popularity of collaborative robots in the future. However, the working scene, the base of manipulator, and the man-robot interaction position are motionless in this research. In future research, a manipulator with moving base and human real-time perceiving for more complex tasks and better interaction needs to be paid attention to. Adding an AGV under the robot and a camera or a sensor on the robot hand could be an effective approach.

The article "Vision-Based Intelligent Perceiving and Planning System of a 7-DoF Collaborative Robot" was published in 2021. Journal: Comput Intell Neurosci.

## Figures and Tables

**Figure 1:** Vision system: the combination of fixed cameras and eye tracker.

**Figure 2:** Details of the human hand structure.

**Figure 3:** The recording of the human operation process. (a–e) Images from RGB cameras. (f–j) Images from the eye tracker.

**Figure 4:** Registration of the visual process. (a) The object, a ball, perceived in the scene. (b) Registration and positioning with the ball in data set.

**Figure 5:** A grasping representation with location, size, and orientation. (a) Grasping rectangle. (b) Bounding box.

**Figure 6:** CNN structure for six-dimensional grasping box planning.

**Figure 7:** CNN structure for three-contact-point planning.

**Figure 8:** Flow chart of the improved RRT based on interpolation.

**Figure 9:** Vision system for operation and environment perceiving. (a) Operation perceiving camera system. (b) Environment perceiving camera system.

**Figure 10:** Environment perceiving vision system for play room table. (a) Perceiving with depth cameras. (b) Perceiving with RGB cameras.

**Figure 11:** Marked hand and robot hand. (a) Hand with marked fingertips. (b) Three-finger robot hand.

**Figure 12:** Registration tests with the objects data set for visual process. (a) Confidence of registration. (b) Accuracy of registration.

**Figure 13:** Grasp position prediction of single objects and combinations. (a–e) Object grasping position. (f) Combination grasping position.

The article "Vision-Based Intelligent Perceiving and Planning System of a 7-DoF Collaborative Robot" was published in 2021. Journal: Comput Intell Neurosci.

**Figure 14:** Grasping point prediction of single selected objects and combinations. (a–e) Selected object grasping position. (f–h) Combination grasping position.

**Figure 15:** Performance of improved RRT with the trajectory planning result and the trajectory only. (a, b) Object 1 trajectory planning. (c, d) Object 2 trajectory planning. (e, f) Object 3 trajectory planning. (g, h) Object 4 trajectory planning. (i, j) Object 5 trajectory planning.

**Figure 16:** Application of IPPS for an unknown bottle in a real environment. (a–d) Trajectory planning. (d–f) Grasping planning. (g–j) Finishing task. (j–m) Man-robot interaction. (m–o) Moving to origin.

**Table 1:** Repeated reverse kinematics accuracy tests on large wrap for index finger (first 4 columns) and thumb (last 3 columns).

Joint	Test 1	Test 2	Test 3	Test 4	Test 5	Standard deviation
*J*0 (degree)	30.038	30.052	30.009	30.088	30.016	0.028238
MCP (degree)	30.057	30.151	30.098	30.139	30.110	0.033075
PIP (degree)	45.120	45.108	45.085	45.177	45.046	0.043069
DIP (degree)	45.072	45.057	45.004	45.105	45.095	0.035556
*J*0 (degree)	179.984	180.081	180.014	180.041	179.990	0.035704
MCP (degree)	30.113	30.018	30.101	30.098	30.052	0.035825
IP (degree)	75.037	75.012	75.022	75.079	75.031	0.023007

**Table 2:** Performance of grasping gesture prediction with CNN.

	Object 1	Object 2	Object 3	Object 4	Object 5
Speed (fps)	20.15	18.33	26.22	18.45	25.12
Success rate (%)	91.5	88.4	93.1	89.0	92.7

**Table 3:** Performance of grasping position prediction with CNN.

	Object 1	Object 2	Object 3	Object 4	Object 5
Error	1.754	2.175	1.540	1.995	1.701
Speed (fps)	55.31	48.09	54.85	50.79	52.70
Success rate (%)	91.4	86.8	92.5	86.6	90.0

**Table 4:** Performance of grasping point prediction with CNN.

	Object 1	Object 2	Object 3	Object 4	Object 5
Error	2.201	2.891	1.885	2.405	2.074
Speed (fps)	43.67	40.55	50.20	41.86	47.04
Success rate (%)	90.0	80.0	95.0	85.0	90.0

**Table 5:** Accuracy of trajectory planning with improved RRT.

Error	*x* (mm)	*y* (mm)	*z* (mm)	*α* (°)	*β* (°)	*γ* (°)
Object 1	3.3	9.5	18.8	0.75	0.21	0.33
Object 2	31.1	40.5	3.4	1.84	0.57	1.88
Object 3	1.2	2.3	3.9	0.20	0.45	0.27
Object 4	8.4	5.0	17.3	0.81	0.19	1.11
Object 5	1.7	3.0	2.5	0.35	0.24	0.71

**Table 6:** Results of improved RRT (first three columns) compared with traditional RRT (last three columns).

	Object 1	Object 2	Object 3	Object 4	Object 5
Error (%)	1.1	2.9	0.4	0.7	0.3
Time (s)	6.08	6.38	5.74	6.45	6.50
Length (mm)	679.5	691.1	668.5	693.0	695.1
Error (%)	2.4	3.7	2.1	1.5	1.7
Time (s)	22.15	24.47	20.87	28.90	30.68
Length (mm)	699.0	707.4	701.5	715.9	709.4

The article "Vision-Based Intelligent Perceiving and Planning System of a 7-DoF Collaborative Robot" was published in 2021. Journal: Comput Intell Neurosci.

**Table 7:** Results of IPPS experiments with objects and combinations in the real environment.

Target object	Attempt 1	Attempt 2	Attempt 3	Attempt 4	Attempt 5
Noodle box	**✓**	**✓**	**✓**	**✓**	**✓**
Coke bottle	**✓**	**✓**	**✓**	**✓**	**✓**
Metal can	**✓**	**✓**	**✓**	**✓**	**✓**
Chips box	**✓**	**✓**	**✓**	**✓**	**✓**
Tea cup	**✓**	**✓**	**✓**	**✓**	**✗**
Coffee bag	**✓**	**✗**	**✓**	**✓**	**✓**
Apple	**✓**	**✓**	**✓**	**✓**	**✓**
Banana	**✓**	**✓**	**✓**	**✓**	**✓**
Mouse	**✓**	**✓**	**✓**	**✗**	**✓**
Stapler	**✓**	**✓**	**✓**	**✓**	**✓**
Tape	**✓**	**✓**	**✗**	**✗**	**✓**
Hammer	**✗**	**✓**	**✓**	**✓**	**✗**
Bowl	**✓**	**✓**	**✓**	**✓**	**✓**
Tissue	**✓**	**✗**	**✓**	**✓**	**✓**
Unknown box	**✓**	**✓**	**✓**	**✓**	**✓**
Unknown bottle	**✓**	**✓**	**✓**	**✓**	**✓**
Unknown bag	**✓**	**✓**	**✗**	**✓**	**✓**
Combination 1	**✓**	**✗**	**✓**	**✓**	**✓**
Combination 2	**✗**	**✓**	**✓**	**✓**	**✓**
Combination 3	**✗**	**✓**	**✗**	**✓**	**✓**

## Data Availability

The data used to support the findings of this study are available from the corresponding author upon request.
